# Assessment of Acoustic Features and Machine Learning for Parkinson's Detection

**DOI:** 10.1155/2021/9957132

**Published:** 2021-08-21

**Authors:** Moumita Pramanik, Ratika Pradhan, Parvati Nandy, Saeed Mian Qaisar, Akash Kumar Bhoi

**Affiliations:** ^1^Department of Computer Applications, Sikkim Manipal Institute of Technology, Sikkim Manipal University, Majitar 737136, Sikkim, India; ^2^Department of Medicine, Sikkim Manipal Institute of Medical Sciences, Sikkim Manipal University, Tadong 737102, Sikkim, India; ^3^Department of Electrical and Computer Engineering, Effat University, Jeddah 22332, Saudi Arabia; ^4^Communication and Signal Processing Lab, Energy and Technology Research Center, Effat University, Jeddah 22332, Saudi Arabia; ^5^Department of Computer Science and Engineering, Sikkim Manipal Institute of Technology, Sikkim Manipal University, Majitar 737136, Sikkim, India

## Abstract

This article presents a machine learning approach for Parkinson's disease detection. Potential multiple acoustic signal features of Parkinson's and control subjects are ascertained. A collaborated feature bank is created through correlated feature selection, Fisher score feature selection, and mutual information-based feature selection schemes. A detection model on top of the feature bank has been developed using the traditional Naïve Bayes, which proved state of the art. The Naïve Bayes detector on collaborative acoustic features can detect the presence of Parkinson's magnificently with a detection accuracy of 78.97% and precision of 0.926, under the hold-out cross validation. The collaborative feature bank on Naïve Bayes revealed distinguishable results as compared to many other recently proposed approaches. The simplicity of Naïve Bayes makes the system robust and effective throughout the detection process.

## 1. Introduction

Parkinson's disease (PD) is an inherent disease among elderly individuals. The disease appears when the dopamine neurons significantly fall in the human brain [1, 2]. The PD symptoms start with voice impairments at its early stage, tremor, and loss of memory, and the subject shows an inability to walk, run, and even perform regular day-to-day duties. The situation worsens at a late age, where the subject suffers huge memory loss and cannot move and lean to perform minor activities. The worst part is that the disease is not curable and not reversible [3], so all efforts have been made to its early detection and preventive measures to suppress its adverse effects. Medical science reveals that Parkinson's disease mainly causes gradual reduction of dopamine hormone in the human brain as this hormone acts as the transmitter of signals among various neurons [4]. Insufficient amount of dopamine hormone leads to nontransmission of signals and various neurorelated disorders and symptoms being started in human beings, and Parkinson's disease is one of them. Symptoms of PD can be nonmotor and motor-related. Nonmotor symptoms include sleep disorder, speech variation, problem in swallowing, and loss of smell, whereas motor symptoms were connected to slow movement, e.g., bradykinesia, tremor, rigidity, and postural instability [5]. These symptoms also vary from patient to patient over different time periods, and the appearance of symptoms is often lately observed by the patient due to the casual ignorance of early symptoms.

The effect of Parkinson's disease varies from person to person, and all the symptoms may not be evident by every PD patient and even may not appear in the same order and same combination. However, subjects suffering from idiopathic rapid eye movement sleep behavior disorder (iRBD) are more prone to PD. Speech changes are the first motor symptom that appears even ten years before the actual diagnosis starts [6]. Therefore, assessing speech signals provides a better scope for detecting chances of Parkinson's in the early stage. For instance, the time domain amplitude of both controls and Parkinson's has been visualized in Figure 1. Each block of Figure 1 represents a subject, where the green color plots represent controls and the red color plots represent the subjects suffering Parkinson's. The subjects' specific plots are generated on the pronunciation of sustaining vowel/a/in Italian language [7].

From Figure 1, the amplitude of Parkinson's subjects appears to be abnormal, where the disorder can be identified. On the other hand, the amplitude of the Non-Parkinson's Disease subject is uniformly in a decreasing trend. The disorder signal of Parkinson's subjects is the dysphonia and hypokinetic dysarthria that a subject suffers at various stages of PD [8]. Dysphonia refers to the inability to produce normal phonation due to impaired functioning of the phonatory system. Reduction of pitch variation often denotes monotonicity and reduces loudness, breathless voice, and tiny speech formation [9]. Approximately 90% of the PD patients are affected by this combined sign of hypokinetic dysarthria [9]. In the context of acoustic voice analysis, it is difficult to identify the slight variation of a sound wave through the naked ears. In such a situation, the power of machine learning techniques can be employed to discriminate Parkinson's from the other signal [10, 11].

As PD is a nonreversible disease, the only option left with the clinical practitioners is to reduce the speed of the effect. In this way, the subject feels confident and cured if the diagnosis process starts early. PD shows only a few symptoms at the early stage on the flip side of the coin, like voice disorder and mild tremors. However, these symptoms also resemble other symptoms of an average person. This is why diagnostic technicians and clinical practitioners are nowadays exploring machine learning and artificial intelligence approaches [12–14] to predict the presence and severity of disease among their subjects.

The main contribution of this article is as follows:

- A collaborative feature bank consisting of seven vocal features has been created from Baseline Features (BF), Vocal Fold Features (VFF), and Time Frequency (TFF) with the help of Correlated Feature Selection (CFS) [15], Fisher Score Feature Selection (FSFS) [16], and Mutual Information-Based Feature Selection (MIFS) [17].
- The traditional Naïve Bayes has been trained and tested on the seven features of the collaborative feature bank, which shows the robustness and effectiveness of our system as compared to other recent approaches of Parkinson's disease detection.

The rest of the article is as follows.  Section 2 deals with literature reviews, Section 3 outlines the materials and methods, and Section 4 briefly discusses the results, followed by a conclusion at Section 5.

## 2. Literature Review

Many recent machine learning techniques, including Naïve Bayes, proved useful in segregating subjects suffering PD from the controls. For instance, Avuçlu and Elen [18] proposed Parkinson's detection through multiple classifiers. Their experiment was conducted on various training and testing instances spanned over 22 vocal features of 195 sound samples. The k-Nearest Neighbor, Random Forest, Support Vector Machine, along with Naïve Bayes, have been used to detect Parkinson's. It has been observed that the Naïve Bayes detects the Parkinson's subjects with 70.26% accuracy with a precision of 0.64. Bourouhou et al. [19] compared many classifiers to predict the presence of Parkinson's among subjects. Their experiment was conducted on 40 subjects comprising 20 Parkinson's and control subjects. The experimental results Naïve Bayes detector revealed a detection accuracy of 65%, the sensitivity of 63.6%, and specificity of 66.6%, respectively. On a similar note, Zhang et al. [20] used Naïve Bayes along with other machine learning techniques to detect Parkinson's disease. Their approach employed signal processing techniques to extract relevant features from the acoustic signal of Parkinson's and control subjects. At the next stage Naïve Bayes, Support Vector Machine (SVM), Logistic Regression (LR), and single and double-layered neural networks have been used to segregate Parkinson's and control subjects. With the 22 vocal features, the Naïve Bayes reveals 69.24% of detection accuracy with a 96.02% of the precision rate. Meghraoui et al. [21] proposed Bernoulli and Multinomial Naïve Bayes (BMNB) on harmonicity, pitch, and pulse features. The BMNB approaches are proved to be a better solution to detect the presence of Parkinson's. A test on 28 samples comes across with a 62.5% detection accuracy on Bernoulli Naïve Bayes (BNB) with 0.375 Mean Squared Error (MSE). Kadiri et al. [22] proposed a method of Parkinson's disease detection using SVM on Single Frequency Filtering Cepstral Coefficients (SFFCC) and Shifted Delta Cepstral (SDC) features exacted from voice signals of Parkinson's and control subjects. The SFFCC + SDC features witnessed 9% of performance improvements as compared to traditional MFCC + SDC features. The traditional SVM on SFFCC + SDC features shows 73.33% detection accuracy with 73.32% F1-score.

Apart from Naïve Bayes, many other supervised techniques, including but not limited to famous deep learning techniques, have been proposed to detect Parkinson's among subjects. Recently Jain et al. [23] proposed a Parkinson's detection method using multiple classifier ensembles. The authors used Synthetic Minority Oversampling Technique (SMOTE) to generate artificial samples for prediction. Their proposed approach on Deep Neural Network (DNN) detects Parkinson's with a detection accuracy of 91.47%. Though the result seems impressive, their approach does not appear practical for many reasons. The authors used the dataset proposed by Sakar et al. [24], and the dataset contains replicated speech information of 252 subjects resulting in 756 instances. Machine learning methods cannot be directly applied to these instances as each subject has three readings of the speech signal. These instances need to be consolidated before the actual classification starts. Moreover, creating a Parkinson's detection system on 754 features is not convincing. The Performance of DNN, as claimed by the authors, may vary on consolidated instances. Further, their system may not be practically effective on synthetic samples generated by SMOTE. Similarly, Polat and Nour [25] use multiple classifiers ensemble to detect Parkinson. The One Against All (OAA) sampling technique plays a pivotal role in the detection process. The Logistic Regression (LR) on OAA samples proved to be a brilliant Parkinson's detector. Multiple supervised classifiers are also used on vocal features selected through Adaptive Grey Wolf Optimization Algorithm (AGWOA) and Sparse Auto Encoder (SAE) [26]. The Naïve Bayes classifier on AGWOA and SAE features reveals a detection accuracy of 72%. In the recent past, decision trees are gaining popularity in biomedical data classification [27]. Classification and Regression Tree (CART) have been used to detect the presence of Parkinson's [28], where the CART detector detects Parkinson's with 75.19% through 8 optimum features of vowel /a/.

## 3. Materials and Methods

### 3.1. Dataset

The idea behind the proposed approach is the feature collaboration to detect Parkinson's disease. For feature collaboration, the Baseline Features (BF), Vocal Fold Features (VFF), and the Time Frequency Features (TFF) about the acoustic signal of both Parkinson's and control patients have been considered. All the BF, VFF, and TFF are extracted from a recent Parkinson's detection database publicly available at the UCI machine learning repository [24], prepared at the Department of Neurology in Cerrahpaşa, Faculty of Medicine, Istanbul. The database contains 752 acoustic features of 252 subjects, including control and Parkinson's. Data is prepared with a 44.1 kHz microphone setting followed by a physician's examination. The sustained phonation of the vowel /a/ was collected from each subject with three repetitions.

The vast 752 features also include 22 VFF, 11 TFF, and 21 BF. These features are extracted using Praat acoustic analysis software [24]. The number of features available under VFF, TFF, and BF of the dataset has been presented in Table 1. Gender-specific control and sick subjects are outlined in Table 2. The detailed characteristics of these features segments and corresponding features can be found at [24, 27].

The Istanbul acoustic database [24] used here comprises 252 subjects, where 64 are controls, and 188 subjects are suffering from Parkinson's. Similarly, the dataset contains vocal information of 122 female (41 controls and 81 Parkinson's) and 130 male subjects (41 controls and 81 Parkinson's).

### 3.2. Features Selection

For effective collaboration, a Features Bank (FB) is created using the best features of BF, VFF, and TFF. The identification of best features has been established through three prominent feature selection techniques [29, 30]— Correlated Feature Selection (CFS) [15], Fisher Score Feature Selection (FSFS) [16], and Mutual Information-based Feature Selection (MIFS) [17]. These feature selection schemes initially ranked the features (based on their contribution towards the classification). They selected the most suitable features from the ranked features (features having the highest contribution towards the classification process). All three CFS, FSFS, and MIFS techniques use distinct proven mechanisms for feature ranking. The CFS calculates correlation among attributes to understand the variable similarity. For two attributes *A*={*a*_1_, *a*_2_, *a*_3_,…, *a*_*n*_} and *B*={*b*_1_, *b*_2_, *b*_3_,…, *b*_*n*_}, CFS calculates correlation *r* as follows:

(1) $$\begin{array}{c} r=\frac{\sum_{i=1}^{n}\left(a_{i}-\bar{a}\right)\left(b_{i}-\bar{b}\right)}{\sqrt{\sum_{i=1}^{n}{\left(a_{i}-\bar{a}\right)}^{2}\sum_{i=1}^{n}{\left(b_{i}-\bar{b}\right)}^{2}}}, \end{array}$$

where $\bar{a}$ = mean of attribute *A* and $\bar{b}$ = mean of attribute *B*. The higher the value of *r*, the more the underlying attributes correlated and the lower the value of *r* the underlying attributes have far deviated from each other. After calculating the correlation score for each attribute, the attributes are arranged in the ascending order of the correlation score. Arranging attributes based on correlation score provides a scope to move the highly uncorrelated attributes to the front and perfectly correlated attributes at the rear, thus supporting the classifiers for enhanced detection. Similarly, FSFS calculates the fisher score of individual features of the underlying Parkinson's dataset. The feature weights are calculated based on the sample size and number of class labels. FSFS are tested for binary and multiclass datasets, but it is widely used for binary datasets [31]; hence, a suitable feature ranker is proposed for the current work. For a given set of features *f*={*f*_1_, *f*_2_, *f*_3_,…, *f*_*p*_} having a set of classes *K*={*k*_1_, *k*_2_, *k*_3_,…, *k*_*c*_}, the fisher score *S* of the feature *f*_*i*_ can be estimated as follows:

(2) $$\begin{array}{c} S=\frac{\sum_{j=1}^{C}n_{j}{\left(\mu_{ij}-\mu_{i}\right)}^{2}}{\sum_{j=1}^{c}n_{j}\rho_{ij}^{2}}, \end{array}$$

where *n*_*j*_ is the number of instances in the *j*^th^ class, *μ*_*i*_ is the mean of the *i*^th^ feature, and *μ*_*ij*_ and *ρ*_*ij*_ are the mean and variance of the *i*^th^ feature and *j*^th^ class, respectively. In this way, the fisher score of each feature of the Parkinson's dataset has been calculated, allowing us to rank the features based on the score accumulated. It should be noted that the fisher score evaluates the score individually; i.e., no two features are taken simultaneously to calculate the feature's score [32]. The individual fisher score proved to be a limitation to identify the feature redundancy. However, since prominent features have been selected iteratively through Naïve Bayes classification, the limitation of identifying feature redundancy will not affect the evaluation process. With a similar guideline of CFS, the MIFS ranking algorithm estimated the relationship among features through mutual information and ranked the features based on the mutual information score of attributes. For any two given attributes *a* and *b* having values {1,…, *p*} and {1,…, *q*}, respectively, a joint probability *π*_*ab*_ ensures the samples of attribute (*a*, *b*) ∈ {1,…, *p*} ×{1,…, *q*}, then the dependency between *a* and *b* can be estimated [17] through mutual information as follows:

(3) $$\begin{array}{c} MI=\sum_{a=1}^{p}\sum_{b=1}^{q}\pi_{ab}\log\frac{\pi_{ab}}{\sum_{b}\pi_{ab}\sum_{a}\pi_{ab}}. \end{array}$$

Like correlation score, mutual information places a crucial role in features ranking. All the three feature ranking algorithms CFS, FSFS, and MIFS can also be extended to select a subset of features. After ranking all ranked feature segments, the ranked features are passed to Naïve Bayes incrementally *one* feature at a time in an iterative fashion. The incremental feature classification allows selecting the suitable number of features from each segment where the Naïve Bayes shows the highest detection accuracy.

In a nutshell, all the three feature selection techniques CFS, FSFS, and MIFS work jointly to identify goodness scores for each attribute of the underlying Parkinson's dataset. The idea behind this incremental feature selection is to select only those attributes which are mainly close to class attributes and not close to each other. However, instead of depending on the practical way of identifying attributes, selecting attributes through incremental classification is emphasized. In a landscape, the incremental feature selection helps to identify potential attributes in the most realistic way. The selected features of BF, VFF, and TFF through CFS, FSFS, and MIFS provide the most relevant collaborative Parkinson's disease detection features. The entire process of Parkinson's detection process has been depicted in Figure 2.

The process of detecting subjects affected with Parkinson's follows three steps; viz., Feature Selection, Feature Collaboration, and Parkinson's Detection. As pointed earlier, in the feature selection stage, the BF, TFF, and VFF are ranked separately using CFS, FSFS, and MIFS techniques. As a result, nine feature blocks are realized. The feature collaboration stage's ranked feature blocks are passed, where Naïve Bayes play a crucial role in suitable feature identification. Features from each ranked feature block are fetched incrementally and sent to Naïve Bayes for classification. This process continues till all features are fetched from each ranked feature block. The incremental features for classification help identify the minimum number of features required to achieve maximum detection accuracy. The number of ranked features for which the maximum amount of detection accuracy has been received are identified. For each feature block, i.e., VFF, TFF, and BF, the best features are identified by comparing all three feature ranking schemes (i.e., CFS, FSFS, and MIFS).

### 3.3. Classification

The ranked features are collaborated and sent to Naïve Bayes for detection of Parkinson's. In this way, the entire detection process relies on a small number of collaborative features; thus, it appears to be a practical method of Parkinson's detection. The detection approach has been developed using the Weka machine learning repository [33, 34]. The implementation settings of the proposed model are outlined in Table 3.

The predictive model of Naïve Bayes uses estimator classes for prediction [35]. The numeric estimator precision values are chosen based on the analysis of the training data. The batch size indicates the desired number of instances to process for batch prediction of testing samples. The supervised discretization option ensures the conversion of numerical attributes to nominal ones. All the attributes remain numerical, so this option has been disabled during the training and testing process.

## 4. Results and Discussion

The results of the proposed work have been analyzed in three broad ways. At the first stage, the efficiency of feature ranking schemes, i.e., CFS, FSFS, and MIFS, has been analyzed. The individual ranking of features per feature selector helps identify the most potential VFF, TFF, and BF segments for effective collaboration. At the second stage, the performance of Naïve Bayes has been evaluated along with many other traditional supervised classifiers in the context of Parkinson's detection. Finally, the proposed collaborative feature-based Parkinson's detection system has been compared against other recent vibrant Parkinson's detection mechanisms.

### 4.1. Collaborative Features Identification

As the first stage of the collaborative Parkinson's detection scheme, a bank of collaborative features is prepared. The detection accuracy of Naïve Bayes on change in the vocal fold, time frequency, and baseline feature through CFS, FSFS, and MIFS ranking has been presented in Figures 3–5, respectively. The classification accuracy of Naïve Bayes was also recorded on original features to understand the power of feature ranking techniques.

It is to note that both the original and the ranked acoustic features are incrementally processed through Naïve Bayes to observe the performance enhancement with a change in the number of features. The performance of Naïve Bayes due to CFS, FSFS, and MIFS shows a satisfactory result as compared to original features. It can be seen from Figure 3 that the CFS shows the highest detection accuracy with just ten features in hand. In contrast, the same Naïve Bayes took 12 original features to produce similar detection accuracy. On the other hand, the three features of the FSFS ranked scheme help the Naïve Bayes attain the same CFS detection accuracy. On a similar note, the Naïve Bayes shows the same detection accuracy with 6 MIFS features. Therefore, all the three CFS, FSFS, and MIFS boost the performance of Naïve Bayes to the peak with the help of 10, 3, and 6 features, respectively. Therefore, the 3 FSFS features have been sent to the feature bank for collaboration.

With a similar guideline, when both the original TFF features and ranked CFS, FSFS, and MIFS features are processed incrementally, only the 3 features of CFS boost the performance of Naïve Bayes exceptionally well up to 75.79%. However, FSFS also boosts the Naïve Bayes' performance but not as that of CFS and MIFS. Both FSFS and MIFS reveal a satisfactory performance improvement with a detection accuracy of 73.4% and 73.81%, respectively. Though the Naïve Bayes took only 1 MIFS feature, the first 3 features of CFS have been sent to the feature bank for collaboration due to the highest detection accuracy.

When the performance of Naïve Bayes is studied, the performance of the classifier due to rankers CFS, FSFS, and MIFS was found to be degraded. Nevertheless, the rankers show a similar result as that of original arrangements with minimal features. In this regard, the Naïve Bayes yields the highest accuracy of 76.59% with 3FSFS features. But instead of FSFS, we prefer to choose 1 CFS ranked baseline feature. The CFS enhances the performance of Naïve Bayes with the same detection accuracy parallel to the original order of features with a lesser number of features. Therefore, the first feature of baseline ranked through CFS ranker has been shortlisted and sent to feature bank for collaboration.

The performance of Naïve Bayes on CFS, FSFS, and MIFS and the original order of VFF, TFF, and BF features have been presented in Table 4. The feature threshold column indicates the minimum number of features identified to produce maximum detection accuracy under the concern settings. So, a total of 3 FRFS ranked vocal fold features. 3 CFS ranked time frequency features and 1 CFS ranked baseline features are identified for feature collaboration.

### 4.2. Performance Analysis of Collaborative Parkinson's Detection

As the first stage of collaborative Parkinson's detection scheme, a bank of 7 collaborative features comprising VFF, TFF, BF has been prepared. Those 7 features have been undergone 10-fold cross validation on Naïve Bayes classifier. The result obtained both for Parkinson's and control subjects has been presented in Table 5.

According to Table 5, the sensitivity of Parkinson's subjects and specificity of control subjects are satisfactory. The specificity of 0.926 for control subjects indicates that the collaborative Parkinson's detection model correctly detects negative results for 92.6% of control subjects who have undergone the test. Similarly, the sensitivity of 0.926 for Parkinson's subjects pointed out that the model will correctly return a positive result for 92.6% of the disease subjects. Similarly, a precision of 0.817 indicates a total of 174 subjects are suffering from Parkinson's out of all the subjects that are predicted as Parkinson's, which is impressive in the context of medical diagnosis. On the other hand, the Receiver Operating Curve (ROC) represents an excellent AUC (>71%). The Precision-Recall Curve (PRC) represents 0.905, which is again in an acceptable range. The ROC and the PRC of subjects predicted as control or Parkinson's have been presented in Figure 6.

According to Figure 6(a), the ROC of both the Control and Parkinson's subjects is entirely satisfactory. The curves are tending nicely towards the true positive rate. The curves claim 76.2% area of the plot both for Controls and Parkinson's subjects. On the other hand, the PRC is convincing for Parkinson's subjects, whereas for the control subjects, the PRC is not convincing (Figure 6(b)).

### 4.3. Performance Comparison with Other State-of-the-Art Models

This section highlights the comparison of the proposed work with other similar classifiers for Parkinson's disease detection. The seven collaborative features used are also passed to the C4.5 decision tree, k-Nearest Neighbor, Logistic Regression, Neural Network, and Random Forest classifiers. The hold-out validation method has been employed to validate the proposed model with other state-of-the-art approaches. In the view of hold-out validation, the training instances are prepared with 30% of the subjects, and the testing instances are 70% of subjects randomly. It is observed that Naïve Bayes on collaborative features excels with 78.97% of detection accuracy with the lowest ever training time. The k-Nearest Neighbor suffers on the collaborative features with the lowest detection accuracy of 67.46%. However, the training time of k-Nearest Neighbor is at par with that of Naïve Bayes. On the other hand, Logistic Regression shows a close performance outcome of Naïve Bayes with a bit of training time of 0.03 s. The detailed performance outcomes of the proposed approach, along with others, are presented in Table 6.

In a subsequent attempt, errors generated by the proposed collaborative Parkinson's detection system have been observed along with peer supervised classifiers. The errors generated by the various classifiers along with collaborative features based on Naïve Bayes represent an inconclusive result. It is because the collaborative PDS shows better results for Mean Absolute Error (MAE). In contrast, it shows at par results with other classifiers in Root Mean Squared Error (RMSE), Relative Absolute Error (RAE), and Root Relative Squared Error (RRSE). The outcome of error matrices such as Mean Absolute Error (MAE), Root Mean Squared Error (RMSE), Relative Absolute Error (RAE), and Root Relative Squared Error (RRSE) have been presented in Table 7.

Similarly, the Naïve Bayes based on collaborative features is also compared with other classifiers through ROC and PRC. The results about the various classifiers have been outlined in Table 8.

In Table 8, Naïve Bayes represents exceptional ROC and PRC Values of 76% and 81%. The results appear to be far better than that of the k-Nearest Neighbor and C4.5 decision tree. The Logistic Regression is the only classifier that closely competes with Naïve Bayes. The ROC and PRC are visually represented for all classifiers, including Naïve Bayes in Figure 7 for control and Parkinson's subjects.

ROC of all the classifiers, including Naïve Bayes, can be seen more towards True Positive Rates. However, C4.5 and k-Nearest Neighbor suffers for controls but shows marginal results for Parkinson's subjects. In addition, with the progression of false positives, k-Nearest Neighbor reveals low true positive rates, and thus, results in low AUC. On the other hand, while evaluating PRC, it is found that Naïve Bayes outperforms with superior precision. Therefore, the proposed collaborative features on Naïve Bayes is a practical approach to Parkinson's detection. At the final stage of analysis, the proposed collaborative features-based Parkinson's detection system has been compared with the current state-of-the-art function-based methods, viz., Avuçlu and Elen [18], Bourouhou et al. [19], Zhang et al. [20], Meghraoui et al. [21], Kadiri et al. [22], Polat and Nour [25], Xiong and Lu [26] and Mekyska et al. [28]. Since our approach is based on a function-based approach, most of the methods taken for comparison belong to function-based approaches such as Naïve Bayes and Support Vector Machine (SVM). The comparison has been conducted in two different sets of performance matrices. At first, the standard detection accuracy has been used for the comparison (Table 9). Finally, the Naïve Bayes based Parkinson's detection mechanisms are compared and analyzed using many other additional performance matrices and are presented in Table 10.

The detection result of five recent Parkinson's disease detection (PDD) schemes has been tabulated in Table 9 along with the proposed collaborative PDD scheme. All these methods used function-based approaches. It has been observed that the proposed collaborative approach claims the highest detection accuracy with the relatively lowest number of vocal features. Though the SVM approach of Kadiri et al. [22] shows 73.32% detection accuracy, which is close to our approach, but at the same time, the number of vocal features used is not clearly highlighted.

A detailed comparison through additional performance measures helps to visualize the capability of the proposed approach over other Naïve Bayes approaches. For this comparison, the Avuçlu and Elen [18] and Bourouhou et al. [19] methods are taken into consideration. According to Table 10, the Avuçlu and Elen [18] method has the highest sensitivity score of 0.949. Therefore, the concerned method indicates that 94.9% of Parkinson's subjects are detected among all the Parkinson's subjects. On the other hand, our proposed PD detection model is more precise with a 0.926 precision rate. In addition, it shows the lowest false positive rate in detecting control subjects as Parkinson's.

## 5. Discussion, Limitations, and Future Works

Like any other detection model, the proposed method also suffers few limitations. The proposed model is based on a voice signal dataset provided by the Department of Neurology in Cerrahpaşa, Faculty of Medicine, Istanbul. The pronunciation ascent of the sustained vowel /a/ is different for different geographical regions. As a result, the model may generate significant false positives or false negatives on the voice signals of subjects of other continents. Therefore, it is essential for further evaluation of other voice signal datasets. As future work, the proposed model can be extended to a graphical user interface mode which must have scope to be trained on varying Parkinson's signal datasets. Gender and age of subjects are other aspects that need a detailed investigation, which the proposed approach lacks. It should be noted that gender and age play a significant role in vocal performance both for control and Parkinson's subjects [36, 37]. An unbalanced dataset age and gender concerning disease pose considerable issues towards the detection process [36–39]. Therefore, the number of participants in the dataset should be balanced based on genders and age for both Parkinson's and control classes. The assessment of gender and age parameters is missing in this research work and will remain a limitation. The disease severity is another factor that allows a detector to determine the stage of the PD. In the future, the proposed work can be modeled to predict the severity of the disease.

A good Parkinson's detection dataset containing acoustic features of the subjects needs to address various factors such as the balance of gender concerning age, microphone quality, noise, the robustness of analysis procedure, number of subjects, disease severity, and influence of medication. Recently, Rusz et al. [40] presented a guideline for speech recording, which can prepare acoustic datasets for Parkinson's detection. The dataset considered here addresses and meets almost all the parameters stated above. However, it still fails to reveal the disease severity, which is a critical issue for any Parkinson's detection system that relies on the dataset used here. Therefore, the proposed work needs to be validated for disease severity prediction, which will make the application practical for clinical use.

Similarly, incorporating event-driven methods may improve the performance of suggested solutions in terms of computational effectiveness, compression, and power consumption [41–44]. Future work considering these aspects may be investigated.

## 6. Conclusion

In this article, a collaborative PDD model has been proposed. The model relies on the vocal fold, time frequency, and baseline features of both control and Parkinson's subjects. These vocal features are first ranked through correlation, fisher score, and mutual information-based feature selection schemes. The ranked features have been passed sequentially to many classifiers where Naïve Bayes evolved as the best classifier for the proposed model. The feature points are also identified based on the highest detection accuracy reported by Naïve Bayes. Relevant features are selected based on these feature points. A total of 7 ranked features has been selected from the vocal fold, time frequency, and baseline feature segments. The detection model based on the 7 ranked features shows promising detection accuracy of 78.97% and precision of 0.926, under the hold-out cross validation. The proposed model has also been compared with other function-based detection models, where our PD detection model proved to be accurate and precise. Finally, an extensive discussion has been carried out regarding the shortcoming and future direction of the proposed Parkinson's detection model.

## Figures and Tables

**Figure 1:** Amplitudes of controls and Parkinson's subjects.

**Figure 2:** The process of collaborative Parkinson's detection.

**Figure 3:** Classification accuracy of Naïve Bayes with change in original features and ranked features on VFF.

**Figure 4:** Classification accuracy of Naïve Bayes with change in original features and ranked features on TFF.

**Figure 5:** Classification accuracy of Naïve Bayes with change in original features and ranked features on BF.

**Figure 6:** (a) Receiver Operating Curve of collaborative Parkinson's detection for Parkinson's and Control subjects. (b) Precision-Recall Curve of collaborative Parkinson's detection for Parkinson's and Control subjects.

**Figure 7:** The receiver operating and precision-recall curves of the collaborative Parkinson's detection for Naive Bayes and its comparison with other supervised learning techniques. (a) Performance comparison, receiver operating curves, on control subjects. (b) Performance comparison, receiver operating curves, on Parkinson's subjects. (c) Performance comparison, precision-recall curves, on control subjects. (d) Performance comparison, precision-recall curves, on Parkinson's subjects.

**Table 1:** Features of Istanbul acoustic dataset.

Features group	Number of features
*Vocal fold features*	
Glottis quotient	3
Glottal to noise excitation	6
Empirical mode decomposition	6
Vocal fold excitation ratio	7
*Time frequency features*	
Voice intensity	3
Bandwidth	4
Formant frequencies	4
*Baseline features*	
Entropy of recurrence period density	1
Detrended fluctuation	1
Entropy of pitch period	1
Harmonicity	2
Variants of jitter	5
Fundamental frequency	5
Variants of shimmer	6

**Table 2:** Gender-specific controls and subjects suffering from Parkinson's in the dataset.

Genders (↓)/Classes (⟶)	Controls	Parkinson's	Total
Female (—)	41	81	122
Male (—)	23	107	130
Total	64	188	252

**Table 3:** Settings used for Naïve Bayes.

Settings	Value
Batch size	100
Use kernel estimator	True
Use supervised discretization	False

**Table 4:** Highest detection accuracy of Naïve Bayes due to ranked acoustic features and original features.

Feature selection techniques	Vocal fold		Time frequency		Baseline	
	Feature threshold	Accuracy	Feature threshold	Accuracy	Feature threshold	Accuracy
CFS	10	76.59	3	75.79	1	75.40
FSFS	3	76.59	2	73.41	3	76.59
MIFS	6	76.59	1	73.81	1	74.60
Original	12	76.59	1	66.67	3	75.40

**Table 5:** Performance of collaborative Parkinson's detection on Naïve Bayes.

Subjects	Sensitivity	Specificity	Precision	F-measure	MCC	ROC area	PRC area
Control	0.391	0.926	0.641	0.485	0.380	0.762	0.514
Parkinson's	0.926	0.391	0.817	0.868	0.380	0.762	0.905

**Table 6:** Detection accuracy and misclassification rate of collaborative Parkinson's Detection using Naïve Bayes and other supervised classifiers.

Classifiers	Number of features	Training time (Sec)	Accuracy (%)	Misclassification rate (%)
C4.5 decision tree	7	0.03	73.81	26.19
k-Nearest Neighbor	7	0.01	67.46	32.54
Logistic Regression	7	0.03	77.38	22.62
Neural Network	7	0.14	75.40	24.60
Random Forest	7	0.21	76.98	23.02
**Naïve Bayes**	**7**	**0.01**	**78.97**	**21.03**

**Table 7:** Error matrices of collaborative Parkinson's detection using Naive Bayes.

Classifier	Attributes	MAE	RMSE	RAE	RRSE
C4.5 decision tree	7	0.33	0.46	86.12	104.99
k-Nearest Neighbor	7	0.33	0.57	86.02	130.45
Logistic Regression	7	0.31	0.40	80.33	91.63
Neural Network	7	0.31	0.42	80.42	96.26
Random Forest	7	0.31	0.40	81.26	92.33
**Naïve Bayes**	**7**	**0.26**	**0.41**	**68.47**	**95.24**

**Table 8:** ROC area and PRC area of collaborative Parkinson's detection using Naive Bayes.

Classifier	Attributes	ROC area	PRC area
C4.5 decision tree	7	0.60	0.69
k-Nearest Neighbor	7	0.56	0.65
Logistic Regression	7	0.75	0.80
Neural Network	7	0.73	0.79
Random Forest	7	0.74	0.78
**Naïve Bayes**	**7**	**0.76**	**0.81**

**Table 9:** Comparison of collaborative Parkinson's detection with other PDS through detection accuracy.

Parkinson's detection methods	Detector	Features	Accuracy (%)
Avuçlu and Elen [18]	Naïve Bayes	22	70.26
Bourouhou et al. [19]	Naïve Bayes	26	65.00
Zhang et al. [20]	Naïve Bayes	22	69.24
Meghraoui et al. [21]	Bernoulli Naïve Bayes	3	62.50
Kadiri et al. [22]	Support Vector Machine	—	73.32
Polat and Nour [25]	Linear Regression	45	77.50
Xiong and Lu [26]	Naïve Bayes	8	72.00
Mekyska et al. [28]	Classification and regression trees	8	75.19
Collaborative PD (proposed)	Naïve Bayes	7	78.97

**Table 10:** Comparison of collaborative Parkinson's detection with other PDS through additional performance measures.

Performance measures	Avuçlu and Elen [18]	Bourouhou et al. [19]	Proposed collaborative PDS
Number of vocal features selected	22	26	7
Balanced detection accuracy	0.699	0.650	0.729
Sensitivity	0.949	0.700	0.817
Specificity	0.448	0.600	0.641
Precision	0.639	0.636	0.926
False negative rate	0.051	0.300	0.183
False positive rate	0.552	0.400	0.359

## Data Availability

The dataset used in this paper is publicly available via the UCI Machine Learning Repository with the labels and link as follows: (a) Parkinson's Disease Classification Data Set (https://archive.ics.uci.edu/ml/datasets/Parkinson%27s+Disease+Classification); (b) Italian Parkinson's voice and speech (https://ieee-dataport.org/open-access/italian-parkinsons-voice-and-speech#files).
